The article "Application Value of the Diagnosis during Early Carcinoma of Upper Digestive Tract Based on Optical Enhanced Endoscopic Technique" was published in 2022. Journal: Comput Math Methods Med.

# Application Value of the Diagnosis during Early Carcinoma of Upper Digestive Tract Based on Optical Enhanced Endoscopic Technique

**DOI:** 10.1155/2022/9587070

**Published:** 2022-07-19

**Authors:** Yinghao Song, Yulei Qu, Lu Li, Mengxuan Xing, Baohui Jia, Yingjie Ma, Yong Zhang

**Affiliations:** ^1^Department of Gastroenterology, People's Hospital of Henan University of Chinese Medicine, Henan University of Chinese Medicine, Zhengzhou, 450000 Henan Province, China; ^2^Department of Gastroenterology, Zhengzhou Central Hospital Affiliated to Zhengzhou University, Zhengzhou University, Zhengzhou, 450000 Henan Province, China; ^3^Xinxiang Medical University, Xinxiang, 453000 Henan Province, China; ^4^Department of Critical Care Medicine, Fourth Affiliated Hospital of Nanchang University, Nanchang University, Nanchang, 330000 Jiangxi Province, China

## Abstract

**Objective:**

The diagnostic value of optical enhanced endoscopy in early cancer of upper digestive tract was studied by comparing the disease accuracy, tumor type, invasion, and various surgical indicators between the two groups.

**Methods:**

188 patients with early upper gastrointestinal cancer treated in our hospital from January 2020 to February 2021 were selected as the research objects. The patients were randomly divided into the observation group and control group with 94 cases in each group.

**Results:**

The accuracy of early detection of early carcinoma of upper digestive tract in the observation group was 94.68% and that in the control group was 76.60%. The accuracy of the observation group was significantly higher than that in the control group, with statistical significance (*P* < 0.05). In the observation group, 36 cases of early gastric cancer, 28 cases of early esophageal cancer, and 30 cases of early colorectal cancer were detected; 25 cases of early gastric cancer, 19 cases of early esophageal cancer, and 28 cases of early colorectal cancer were detected; 26 cases of early carcinoma of upper digestive tract infiltration were detected; and 68 cases were not detected, and the detection rate was 27.66%, which was higher than 9.57% in the control group, and the difference was statistically significant (*P* < 0.05). After different methods of treatment, no death occurred in all patients. Except for the operation time, the surgical indexes of the observation group were better than the control group, the difference was statistically significant (*P* < 0.05).

**Conclusion:**

Optical enhanced endoscopic technique had obvious effect in the diagnosis of patients with early cancer of upper digestive tract, it was helpful to improve the clinical detection rate of early carcinoma of upper digestive tract and had certain diagnostic ability for the invasion depth of early cancer of high upper gastrointestinal tract, which was conducive to the detection of clinical invasion lesions and had high clinical promotion and application value.

The article "Application Value of the Diagnosis during Early Carcinoma of Upper Digestive Tract Based on Optical Enhanced Endoscopic Technique" was published in 2022. Journal: Comput Math Methods Med.

## 1. Introduction

Upper gastrointestinal cancer is one of the most common malignant tumor diseases in clinical practice. According to relevant survey data, with the continuous change of people's lifestyle and dietary structure in recent years, the incidence of upper digestive tract cancer is increasing year by year, which has caused serious impact on the life and health safety of residents [1, 2]. For a long time in the past, many scholars have studied the risk factors of upper gastrointestinal cancer, including smoking, drinking, eating habits, genetics, and infection, which are recognized as the risk factors of upper gastrointestinal cancer [3, 4]. The cancers of the upper digestive tract mainly include gastric, esophageal, and duodenal cancers, which mainly refer to lesions confined to the mucosa or submucosa with or without lymph node metastasis [5]. In addition, due to the extremely insidious nature of upper gastrointestinal cancer in the early stage of its onset, patients generally have no significant clinical symptoms [6]. Therefore, the effective diagnosis of early carcinoma of upper digestive tract is particularly important, and it is also the focus of clinical attention. At present, the main method commonly used in clinical early digestive tract cancer is white light endoscopy, but white light endoscopy is prone to misdiagnosis and missed diagnosis. Optical enhanced endoscopy can make up for this deficiency. Optical enhanced endoscopy has a high detection rate for early digestive tract tumors, which is helpful to assist doctors in early treatment of patients [7, 8]. Optical enhanced endoscopy is a new type of electronic staining endoscopy. Its principle is to enhance the tumor surface structure and blood vessel shape through narrow-band imaging to achieve the observation effect of the tumor, so as to achieve the optical diagnosis of the tumor [9, 10]. The optical enhanced endoscopic technique has the characteristics of simple operation and high accuracy, which can magnify the observation of lesions, improve the conformity with pathological diagnosis, and evaluate the risk of lesions [11, 12].

In this study, 188 cases of early carcinoma of upper digestive tract in our hospital were selected to compare and analyze the application value of optical enhanced endoscopic technique and ordinary high-purity light endoscopy in the identification of upper digestive tract early cancer.

This study consists of four sections.

The article "Application Value of the Diagnosis during Early Carcinoma of Upper Digestive Tract Based on Optical Enhanced Endoscopic Technique" was published in 2022. Journal: Comput Math Methods Med.

Section 2 shows the “materials and methods,” which introduces the basic information of the samples, the sampling methods, and the determination of key indicators.

Section 3 is the comparison results of the two groups. This section compares the two groups according to the three indicators (accuracy, types and infiltration of cancer, and surgical indexes) and obtains the comparison results.

Section 4 is the discussion, and the relevant results are discussed according to the data comparison in Section 3.

Section 5 is the conclusion. This section summarizes the research results of the full text, puts forward the value of this study, and points out the shortcomings of this study.

## 2. Materials and Methods

### 2.1. General Information

A total of 188 patients with early carcinoma of upper digestive tract admitted to our hospital from January 2020 to February 2021 were selected as the research objects.

Inclusion criteria are as follows: ① age ≥ 18 years old, ② the patient had developed the clinical features of early cancer, ③ knowing own illness, ④ the early carcinoma of upper digestive tract was confirmed by histologic biopsy, and ⑤ no relevant antitumor therapy was received before admission.

Exclusion criteria are as follows: ① pregnant women; ② serious diseases of the heart, liver, or kidney; ③ unable to communicate normally or combined with neurological diseases; ④ complicated with other systemic malignancies; and ⑤ other unsuitable candidates.

They were divided into the observation group and control group, with 94 cases in each group. There was no significant difference in clinical data between the two groups, which was comparable (*P* > 0.05). General information of the two groups is shown in Table 1.

### 2.2. Methods

#### 2.2.1. Endoscopy

The control group was diagnosed by ordinary high-purity light endoscopy. The observation group underwent optical enhanced endoscopic technique, and the specific contents were as follows: 30 ml of 1.0% water suspension of dimethicone oil powder was taken orally 30 min before endoscopy, and dacronin hydrochloride gum slurry was given orally for pharyngeal anesthesia 10 min before examination [13]. The observation group was treated with general anesthesia, and then, the morphology, surface microstructure, boundary, and microvascular conditions of the lesions were observed. First, the depth and scope of the lesion were determined by the professional doctor using the optical enhanced endoscope, and the mark was made at the place 5 mm away from the edge of the lesion. Then, submucosal injection was performed on the outside of the mark to make the lesion bulge and separate from the original muscle layer of the patient. The mucosa and submucosa of the lesion were cut along all the mark points. Finally, the tissue at the lesion site was removed and the bleeding and perforation were treated. All endoscopic operations were completed independently by the same professional physician in our hospital.

The article "Application Value of the Diagnosis during Early Carcinoma of Upper Digestive Tract Based on Optical Enhanced Endoscopic Technique" was published in 2022. Journal: Comput Math Methods Med.

#### 2.2.2. Pathological Diagnosis

After the observation of the two groups, a part of the tissue was taken for biopsy, and the pathological biopsy tissue was placed in 10% formalin solution for fixation, and the pathological tissue sections were stained with HE [14]; pathological diagnosis was made by 2 experienced physicians from the Department of Pathology in our hospital. The pathological diagnostic criteria are as follows [15]:

1. Normal: the cytoplasm of mature squamous epithelial cells is rich and clear, and scattered lymphocytes and compressed nuclei are occasionally seen
2. Spinous layer thickening: normal squamous epithelial cells, but thickness ≥ 0.5 mm
3. Inflammation: the papilla of lamina propria grows to the upper third of the epithelium, and the proliferation of basal cells is greater than 15% of the total epithelial thickness. The epithelium was infiltrated by neutrophils or eosinophils. Lamina propria is densely infiltrated by mononuclear inflammatory cells or neutrophils
4. Basal cell hyperplasia: normal epithelium with thickening of basal region and thickness greater than 15% of total epithelial thickness. No extension or other abnormalities of the lamina propria papillae
5. Atypical hyperplasia of squamous epithelium: abnormal nuclear atypia or loss of normal cell polarity and mild atypical hyperplasia involving the lower 1/3 of the epithelium. Moderate atypical hyperplasia involving the upper, middle, and lower epithelial layers, but not involving or infiltrating the whole layer, is called severe atypical hyperplasia

### 2.3. Observational Index

We observe the accuracy of disease, the types and infiltration of cancer, and various surgical indexes of the two groups.

1. Accuracy: number of confirmed cases, number of unconfirmed cases, and accuracy
2. Types and infiltration of cancer: the types of cancer were early gastric cancer, early esophageal cancer, and early colorectal cancer. The infiltration was divided into infiltration and noninfiltration, and the infiltration rate was calculated
3. Surgical indexes: duration of operation, amount of blood loss, length of hospital stay, and treatment cost

### 2.4. Statistical Method

SPSS 18.0 statistical software was used for analysis. Measurement data was expressed as *x* ± *s*. The *t*-test was used for comparison between groups, and the count data was expressed as rate. The *χ*^2^ test was used for comparison between groups, and *P* < 0.05 was considered statistically significant.

The article "Application Value of the Diagnosis during Early Carcinoma of Upper Digestive Tract Based on Optical Enhanced Endoscopic Technique" was published in 2022. Journal: Comput Math Methods Med.

## 3. Results

This section is the comparison results of the two groups. This section compares the two groups according to the three indicators (accuracy, types and infiltration of cancer, and surgical indexes) and obtains the comparison results.

### 3.1. Results of Accuracy

The accuracy of early detection of early carcinoma of the upper digestive tract in the observation group was 94.68% and that of the control group was 76.60%. Results of accuracy are shown in Table 2.

The observation group was diagnosed through the optical enhanced endoscopic technique, and the detection results of the observation group is shown in Figure 1.

The observation group was diagnosed by ordinary high-purity light endoscopy, and the detection results of control group is shown in Figure 2.

### 3.2. Results of Types and Infiltration of Cancer

In the observation group, 36 cases of early gastric cancer, 28 cases of early esophageal cancer, and 30 cases of early colorectal cancer were detected. In the control group, 25 cases of early gastric cancer, 19 cases of early esophageal cancer, and 28 cases of early colorectal cancer were detected. In the observation group, 26 cases of early carcinoma of upper digestive tract infiltration were detected and 68 cases were not detected, and the detection rate was 27.66%. Results of types and infiltration of cancer are shown in Table 3.

### 3.3. Results of Surgical Indexes

After different methods of treatment, no death occurred in all patients. Except for the operation time, the observation group was higher than the control group. Results of surgical indexes are shown in Table 4.

## 4. Discussion

Cancer of the upper digestive tract has become one of the most important cancers in China. The incidence rate and mortality of cancer of the upper digestive tract are among the highest in China. In 2008, the incidence rate of gastric cancer and esophageal cancer in the national cancer registration areas was 26.58/100000 and 16.24/100000, respectively [16]. Early cancer of the digestive tract can be divided into several types, including esophagus, colorectal, and stomach [17]. Early screening of upper digestive tract cancer and early treatment of upper digestive tract cancer to the early stage or before the occurrence of cancer are extremely effective measures to reduce the incidence of upper digestive tract cancer and control the progress of upper digestive tract cancer [18]. Early esophageal cancer refers to the esophageal cancer in which the invasion depth of the focal area of the patient has reached the mucosal layer, but there is no lymphatic metastasis [19]. Early colorectal cancer refers to the infiltration depth of the patient's focal area to the corresponding mucosal layer or submucosa. Gastric early cancer is also the depth of the lesion reached the corresponding mucosa or submucosa. Compared with white light endoscopy, the withdrawal time of optical enhanced endoscopy is similar, but under the influence of intestinal preparation, this is the advantage of optical enhanced endoscopy compared with other electronic stained endoscopes [20, 21]. Among the above 3 types of cancer, only esophageal cancer was related to the presence or absence of lymphatic metastasis [22]. Under normal circumstances, early carcinoma of upper digestive tract has no obvious clinical manifestations, and the external morphology of the lesions does not change significantly at the beginning of the disease. Patients often do not pay enough attention to it, which delays treatment time, and its diagnostic accuracy is also low in clinical practice. Upper digestive tract cancer screening enables more asymptomatic patients with upper digestive tract cancer to receive corresponding treatment as soon as possible, improves the current traditional cancer treatment mode, and advances the treatment of cancer before the deterioration of the disease, so as to improve the survival rate and quality of life of patients with upper digestive tract cancer [23, 24]. The optical enhanced endoscopic technique uses the concept of optical magnification to magnify it to 80~170 times, which is more direct than high-definition endoscopy [25]. Generally combined with electronic endoscopic staining and mucosal staining, the optical enhanced endoscopic technique can be used for close observation of the small vessels and structures on the mucosal surface of the digestive tract, and the lesions of the mucosa can be directly observed. This technique has a high sensitivity and recognition for intraepithelial neoplasia and gastric mucosal and intestinal metaplasia. Optical enhanced endoscopy has high diagnostic efficiency in real-time diagnosis and differentiation of pathological types of colorectal micropolyps and can reach the broad value of “discovery -retention” and “resection-discard” strategies of electronic staining endoscopy developed by ASGE for micropolyps [26]. The optical enhanced endoscopic technique uses the white light filter and filter calculation of the light source to obtain the narrow band spectrum, through the careful observation of the patient's lesion fine structure and imaging [27, 28]. In addition, electronic endoscopic staining, amplification technology, and mucosal staining can be used to further determine the depth of infiltration of early esophageal cancer. Optical enhanced endoscopy has good interobserver consistency both with and without magnification [29].

The article "Application Value of the Diagnosis during Early Carcinoma of Upper Digestive Tract Based on Optical Enhanced Endoscopic Technique" was published in 2022. Journal: Comput Math Methods Med.

The results of this study found that the accuracy of early detection of early carcinoma of the upper digestive tract in the observation group was 94.68% and that in the control group was 76.60%. 36 cases of early gastric cancer, 28 cases of early esophageal cancer, and 30 cases of early colorectal cancer were detected in the observation group. In the control group, 25 cases of early gastric cancer, 19 cases of early esophageal cancer, and 28 cases of early colorectal cancer were detected. In the observation group, 26 cases of early carcinoma of upper digestive tract infiltration were detected, and 68 cases were not detected, and the detection rate was 27.66%. After different methods of treatment, no death occurred in all patients.

## 5. Conclusion

The optical enhanced endoscopic technique had an obvious effect in the diagnosis of patients with early cancer of the upper digestive tract; it was helpful to improve the clinical detection rate of early carcinoma of upper digestive tract and had certain diagnostic ability for the invasion depth of early cancer of high upper gastrointestinal tract, which was conducive to the detection of clinical invasion lesions, and had high clinical promotion and application value. However, the technology of optical enhanced endoscopy has high technical requirements for medical technicians. The operation team should be equipped with experienced doctors to reduce the false detection rate. At the same time, the diagnosis of early digestive tract cancer under optical contrast-enhanced endoscopy must be strictly combined with pathological diagnosis to get the correct diagnosis results.

## Figures and Tables

**Figure 1:** Detection results of the observation group.

**Figure 2:** Detection results of the control group.

**Table 1:** General information of the two groups.

Groups	Control group	Observation group	*P*
Cases	94	94	
Gender			
Male	45	48	>0.05
Female	49	46	
Age (average)	46.17 ± 11.25	46.56 ± 11.23	>0.05
Clinical manifestation			
Belching	24	20	>0.05
Abdominal distension	16	20	
Acid reflux	28	26	
Gasteremphraxis	26	28	
Inspection			
Gastroscopy	46	49	>0.05
Enteroscopy	48	45	

**Table 2:** Results of accuracy.

Groups	Cases	Confirmed	Unconfirmed	Accuracy (%)
Control group	94	72	22	76.60
Observation group	94	89	5	94.68
*χ* ^2^				25.741
*P*				<0.05

**Table 3:** Results of types and infiltration of cancer.

Groups	Cases	Types of cancer			Infiltration		
		Early gastric cancer	Early esophageal cancer	Early colorectal cancer	Infiltration	Noninfiltration	Infiltration rate
Control group	94	25	19	28	9	85	9.57%
Observation group	94	36	28	30	26	68	27.66%
*χ* ^2^		5.624			4.816		
*P*		<0.05			<0.05		

The article "Application Value of the Diagnosis during Early Carcinoma of Upper Digestive Tract Based on Optical Enhanced Endoscopic Technique" was published in 2022. Journal: Comput Math Methods Med.

**Table 4:** Results of surgical indexes.

Groups	Cases	Duration of surgery (min)	Amount of blood loss (ml)	Length of hospital stay (d)	Treatment cost (ten thousand yuan)
Control group	94	125.36 ± 13.25	125.22 ± 18.14	8.40 ± 2.36	2.15 ± 0.18
Observation group	94	80.15 ± 20.04	85.31 ± 12.30	4.18 ± 1.49	1.37 ± 0.11
*t*		8.038	14.325	18.142	55.634
*P*		<0.05	<0.05	<0.05	<0.05

## Data Availability

The data used to support the findings of this study are included within the article.
